The article "Study to compare the effect of casirivimab and imdevimab, remdesivir, and favipiravir on progression and multi-organ function of hospitalized COVID-19 patients" was retracted in 2023. Reasons: duplicate publication; overlap with earlier publications.

# Study to compare the effect of casirivimab and imdevimab, remdesivir, and favipiravir on progression and multi-organ function of hospitalized COVID-19 patients

**DOI:** 10.1515/med-2023-0768

**Published:** 2023-08-09

**Authors:** Sahar K. Hegazy, Samar Tharwat, Ahmed H. Hassan

**Affiliations:** Clinical Pharmacy Department, Faculty of Pharmacy, Tanta University, Tanta, PC: 31511, Egypt; Rheumatology and Immunology Department, Faculty of Medicine, Mansoura University, Mansoura, PC: 35511, Egypt; Clinical pharmacy Department, Mansoura University Hospital, Mansoura, PC: 35511, Egypt

**Keywords:** antivirals, casirivimab and imdevimab, COVID-19, favipiravir, remdesivir

## Abstract

Coronavirus disease 2019 (COVID-19) caused a progress in research to find a solution to this pandemic. Also, various advances in pharmacotherapy against COVID-19 have emerged. Regarding antiviral therapy, casirivimab and imdevimab are antibodies combination against COVID-19. Standard antiviral therapy against COVID-19 includes remdesivir and favipiravir. The objectives were to compare progression and multi-organ function of hospitalized COVID-19 patients between these three antiviral groups. 265 COVID-19 hospitalized patients were included in this study and were divided into 3 groups (1:2:2), respectively, Group (A): casirivimab and imdevimab, group (B): remdesivir, and group (C): favipiravir. The design of the study is a single blind non-randomized controlled trial. This study is a phase IV clinical trial (post-marketing study). The duration of the study was about 6 months after receiving the ethical approval. Casirivimab and imdevimab achieved less case progression as presented by lower World Health Organization scale (*P* < 0.05 in comparing group A with B and C) and better multi-organ functions as presented by lower Sequential Organ Function Assessment score (*P* < 0.05 in comparing group A with B and C) than remdesivir and favipiravir. From all these results, it is concluded that Group A (casirivimab and imdevimab) produces better outcomes than B (remdesivir) and C (favipiravir) intervention groups.

## 1 Introduction

### 1.1 Coronavirus disease 2019 (COVID-19) overview and classification

COVID-19 is an infectious disease caused by sever acute respiratory syndrome-corona virus 2 (SARS CoV-2) that has affected a lot of human beings all over the world with high mortality rate [1]. COVID-19 infection has been classified [2] as:

Mild: Individuals who have any of the various signs and symptoms of COVID-19 without respiratory symptoms (e.g., fever, cough, sore throat, malaise, headache, muscle pain, nausea, vomiting, diarrhea, loss of taste, and smell) but not having dyspnea, shortness of breath, or abnormal chest imaging.

The article "Study to compare the effect of casirivimab and imdevimab, remdesivir, and favipiravir on progression and multi-organ function of hospitalized COVID-19 patients" was retracted in 2023. Reasons: duplicate publication; overlap with earlier publications.

Moderate: Individuals who show evidence of lower respiratory disease during clinical assessment or imaging, and who have an oxygen saturation (SpO_2_) ≥94% in room air at sea level.

Severe: Individuals suffer from lower respiratory disease with saturation pressure of oxygen (SpO_2_) <94% in room air at sea level, a ratio of arterial partial pressure of oxygen to fraction of inspired oxygen (PaO_2_/FiO_2_) <300 mmHg, respiratory frequency >30 breaths/min, or lung infiltrates >50%.

Critical: Individuals have respiratory failure, septic shock, and/or multiple organ dysfunctions.

Covid-19 crisis causes a progress in research to find a solution to this pandemic. Also, various advances in pharmacotherapy against COVID-19 have emerged [3].

### 1.2 Standard and controversial antivirals used in treatment of COVID-19 (remdesivir and favipiravir)

Remdesivir has been approved by Food and Drug Administration (FDA) for treatment of mild, moderate, severe, and critical hospitalized COVID-19 patients [4]. Other drugs have shown controversial antiviral activity including favipiravir, hydroxychloroquine, ivermectin, nitazoxanide, and ribavirin. Favipiravir was selected from all other investigational antiviral agents, as it is the most investigational antiviral agent used for COVID-19 in Egypt.

Favipiravir has become a standard antiviral drug. Favipiravir is used for treatment of mild and moderate COVID-19 outpatients [5].

### 1.3 Advances in immunotherapy for treatment of COVID-19

Immunotherapy to target virus antigen has been developed [6]. Figure 1 shows two types of immunotherapies, active and passive immunotherapies. In active immunotherapy, body produces antibodies against virus as vaccination. Passive immunotherapy involves direct administration of antibodies to act specifically against virus or administration of product containing antibodies like plasma [6].

**Figure 1:** Immunization approaches against COVID-19 [6].

There are three targets for these antibodies to work as antiviral including antibodies that prevent the virus entry, antibodies that inhibit the virus replication, and antibodies that stop the immune system response.

Table 1 includes various types of antibodies under investigation for treatment of COVID-19 and their targets [6].

**Table 1:** Antibody candidates against SARS-CoV-2 under investigation by pharmaceutical companies [6]

Antibody	Mechanism	Company	Stage of study/identification method
Gimsilumab	Anti GM-CSF monoclonal antibody	Roivant Sciences	In clinical stage for inflammation and rheumatic disease. Prioritized in clinical trial for SARS-CoV-2
Lenzilumab		Humanigen Inc.	Currently in clinical stage for leukemia and lymphoma
Canakinumab (Ilaris®)	IL-1β inhibitor	Novartis	In clinical stage for several inflammatory diseases including arthritis, periodic fever, and lung cancer;Repurposed by Novartis for COVID-19
Secukinumab (Cosentyx®)	IL-17 inhibitor	Novartis	In clinical stage for several autoimmune diseases including psoriasis; Repurposed by Novartis for COVID-19
TZLS-501	Fully human monoclonal antibody targeting the receptor of IL-6, it binds to both membrane-bound and soluble forms of IL-6R, and rapidly depletes the circulating levels of IL-6 in blood	Tiziana Life Sciences and Novimmune	Preclinical stage
ALT-100	Neutralizes circulating NAMPT	Aqualung Therapeutics Corp.	Preclinical stage
Pritumumab	Fully human IgG antibody targeting vimentin	Nascent Biotech Inc.	Received FDA approval for several carcinoma; Research began for COVID-19
Leronlimab (PRO140)	Antagonizes CCR5 on T-cells and prevents viral entry	CytoDyn	A 10-patient clinical study against COVID-19; Initially developed against HIV; in clinical trial for HIV and breast cancer
		
BDB-1	Anti C5a	Beijing Defengrei Biotechnology	Beijing Defengrei Biotechnology passes the phase II of clinical trial
IFX-1		InflaRx	InflaRx received approval for starting the clinical trial in Netherlands
Antibody cocktail including REGN3048 and REGN3051	Fully human multivalent antibodies against the spike protein isolated from genetically modified mice or recovered COVID-19 patients	Regeneron	Phase 1 clinical trial for Middle East Respiratory Syndrome (MERS) completed last yearClinical trial for SARS-CoV

The article "Study to compare the effect of casirivimab and imdevimab, remdesivir, and favipiravir on progression and multi-organ function of hospitalized COVID-19 patients" was retracted in 2023. Reasons: duplicate publication; overlap with earlier publications.

### 1.4 Casirivimab and imdevimab as antibodies cocktail against COVID-19

The point of research is antibodies cocktail including REGN3048 and REGN3051 that refers to two monoclonal antibodies REGN3048 (casirivimab), and REGN3051 (imdevimab) which prevent viral entry into human cells through the angiotensin-converting enzyme 2 receptor [7,8], and have shown an antiviral activity and need for further investigation to prove their benefit in COVID patients [9].

Previous study [9] that was conducted on REGN3048 and REGN3051 ((REGN-COV2 [casirivimab and imdevimab]) has mentioned that efficacy of both these antibodies cocktail is confirmed in COVID-19 outpatients’ treatment in both low (2.4 g of REGN-COV2), or high (8.0 g of REGN-COV2) dose when compared to placebo.

Efficacy is measured as virologic efficacy: Time-weighted change in viral load from baseline through day 7 (log10 scale) in patient, and clinical efficacy: Symptoms offset on day 7 and percentage of patients with one or more medically attended visits.

This previous study [9] proved that efficacy is more obvious in seronegative outpatients (whose immune response is not effective yet to produce antibodies against virus) and with high baseline viral load outpatients.

The article "Study to compare the effect of casirivimab and imdevimab, remdesivir, and favipiravir on progression and multi-organ function of hospitalized COVID-19 patients" was retracted in 2023. Reasons: duplicate publication; overlap with earlier publications.

Now, data [10] are available for these new antibodies’ combination. The US FDA has allowed an Emergency Use Authorization (EUA) for this combination in the post-exposure prophylaxis and treatment of mild and moderate COVID-19 outpatients with positive PCR results of direct SARS-CoV-2 viral testing, and patients at high risk for progression to severe COVID-19 requiring hospitalization or causing death.

In contrast, REGN3048 and REGN3051 are still not authorized for use in patients who require oxygen therapy due to COVID-19, who require an increase in baseline oxygen flow rate due to COVID-19 in those on chronic oxygen therapy due to underlying non-COVID-19 related comorbidity, and who are hospitalized due to COVID-19 [10].

Now, casirivimab and imdevimab are investigational antibodies, serious and unexpected adverse effects can occur that were not previously reported with their use [10]

These antibodies combination follows linear pharmacokinetics after its single intravenous doses with half-life of about 25–37 days for both antibodies. Regarding elimination, this combination is not metabolized by liver cytochrome enzymes, and not excreted by kidneys [10].

Limitations of previous study include not using many of the clinically relevant outcomes like mortality rate, study performed on non-hospitalized patients only and not including hospitalized patients (trial is done only on outpatients and not inpatients), and not studying the long-term effects of antiviral efficacy in lowering viral load on inflammatory markers.

This research is an extension of a published research article [11].

## 2 Aim of the study

The objectives of this study were to compare case progression as presented by World Health Organization (WHO) scale and multi-organ function as presented by Sequential Organ Function Assessment (SOFA) score in hospitalized COVID-19 patients between the three antiviral groups.

## 3 Patients and population

265 COVID-19 hospitalized patients were included in this study and were divided into 3 groups (1:2:2): group A received Antibodies cocktail (casirivimab and imdevimab), group B received remdesivir, and group C received favipiravir [11].

Population in this study were patients hospitalized in isolation hospital Mansoura university.

A computer file containing a written informed consent from included patients was provided. Paper was not a tool for providing agreement by patients or their relatives to avoid transmission of infection.

### 3.1 Inclusion criteria

weight not less than 40 kg, PCR- confirmed patients to be positive before inclusion, age more than 12 years old, and moderate, sever, or critical COVID-19 disease as defined by WHO [11].

The article "Study to compare the effect of casirivimab and imdevimab, remdesivir, and favipiravir on progression and multi-organ function of hospitalized COVID-19 patients" was retracted in 2023. Reasons: duplicate publication; overlap with earlier publications.

### 3.2 Exclusion criteria

Current use of controversial antiviral therapy (hydroxychloroquine, ivermectin, nitazoxanide, oseltamivir, acyclovir, ribavirin, lopinavir/ritonavir, sofosbuvir, daclatasvir, simeprevir, azithromycin), prior use of standard antiviral therapy (remdesivir or favipiravir), history of hypersensitivity or infusion related reactions after administration of monoclonal antibodies, and patients expected to die within 48 h [11].

### 3.3 Interventions

Population, that were included in this study, were assigned into three groups with 1:2:2 ratios to receive either antibodies combination, remdesivir, or favipiravir as shown in Figures 2 and 3.

**Figure 2:** Assignment of the included COVID cases to their groups.

**Figure 3:** Frequency of interventions in included patients.

Group A patients received REGN3048 and REGN3051(antibodies cocktail, casirivimab and imdevimab) in low-dose regimen of 1.2 g (1,200 mg of combined antibodies) diluted in 250 mL 0.9% sodium chloride solution as single IV infusion over 30–60 min.

Group B patients received remdesivir:

Day 1 (loading dose): 200 mg (two 100 mg vials) diluted in 500 mL 0.9% sodium chloride solution as infused IV over 60 min.

Days 2–5 or days 2–10 (maintenance dose): 100 mg (one 100 mg vial) in 250 mL 0.9% sodium chloride solution as infused IV over 30 min.

Group C patients received favipiravir:

Day 1 (loading dose): 1,600 mg (8 tablets) or 1,800 mg (9 tablets) orally or in Ryle tube/12 h

Days 2–5 or days 2–10 (maintenance dose): 600 mg (3 tablets) or 800 mg (4 tablets) orally or in Ryle tube/12 h

Patients received standard care guided by Egyptian COVID-19 treatment guidelines.


**Consent to participate**: The study was performed in accordance with the Helsinki Declaration of 1964, and its later amendments; All subjects provided informed consent to participate in the study; Written informed consent was obtained from all participants; Written informed consent was obtained from parent/guardian of each participant under 18 years of age; The authors declare that they followed their institutions’ protocols to access the patient’s data and that was done with the unique purpose of the scientific investigation and scientific disclosure.

## 4 Materials and methods

Design of the study was a single blind non-randomized controlled trial. This study was phase IV clinical trial (post-marketing study) to evaluate efficacy of new pharmaceutical products. The duration of the study was about 6 months. Longitudinal model and correlation structure had been used in this research [11].

The article "Study to compare the effect of casirivimab and imdevimab, remdesivir, and favipiravir on progression and multi-organ function of hospitalized COVID-19 patients" was retracted in 2023. Reasons: duplicate publication; overlap with earlier publications.

We used PubMed search tool to find clinical studies that were performed to test the efficacy of the developed immunotherapy in the treatment of COVID-19 with about 4,000 results with focusing on antibodies developed as antiviral against COVID-19 obtaining only 70 results from which REGN-COV2, a neutralizing antibody cocktail is selected with its only one clinical study up to now (REGN-COV2, a Neutralizing Antibody Cocktail, in Outpatients with Covid-19) which is published in New England Journal of Medicine on January 21, 2021.

Another resource, used to obtain data, was fact sheet for health care providers- EUA OF casirivimab and imdevimab which provides clinical data about the use of these antibodies cocktail [11]. Endnote citation software was used for citation of references.

Informed consent was obtained from each patient included in the study. The study protocol conforms to the ethical guidelines of the 1975 Declaration of Helsinki, as reflected in a prior approval by the institution’s human research committee.

The research protocol was approved by IRB, faculty of medicine, Mansoura University, MS21.11.1737, Research ethics committee, faculty of medicine, Tanta University, 35039/11/21, and Research ethics committee, ministry of health, Egypt, 10-2022/18.

Registry name and registration number: Clinicaltrials.gov, NCT05502081.

## 5 Outcomes

Clinical outcomes measured before and during intervention include: COVID19 WHO disease progression score [12] from day 0 to day 28, and SOFA score [13] on day 0, 3, 7, 14, and 28.

In addition to clinical outcomes measured after intervention, patients’ characteristics (age and gender) were recorded at the time of admission.

Duration of research was about 6 months from November 2021 to April 2022 [11].

## 6 Statistical analysis and sample size

Categorical variables were presented as proportion and percent. Continuous variables were presented as mean (standard deviation) for parametric data or as a median (25th–75th percentile) for non-parametric data [11].

Regarding baseline characteristics, Kruskal–Wallis or ANOVA test (depending on the type of data and the continuous data distribution [normal or not]) was used to compare these characteristics between the study groups. We reported the *P*-value for our statistical tests with the level of statistical significance as *P*-value ≤0.05 [11].

In case of existing differences in some baseline characteristics, logistic regression would be performed. This allowed studying the effect of these variables on the primary outcomes of the study to exclude the effect of these confounding variables and to ensure that the effect on the outcomes is due to interventions [11].

The article "Study to compare the effect of casirivimab and imdevimab, remdesivir, and favipiravir on progression and multi-organ function of hospitalized COVID-19 patients" was retracted in 2023. Reasons: duplicate publication; overlap with earlier publications.

Regarding the outcomes, we compared WHO scale, and SOFA score using the Kruskal–Walli’s test, with the reported *P*-value [11].

### 6.1 Sample size

A total sample size of 246 patients would achieve at least 80% power to detect a risk difference of 0.2 (20%) in the WHO scale and SOFA score with a significance level (*α*) of 0.05 and 95% confidence level using the ANOVA or Kruskal–Wallis test of independent proportion in G*Power software. To compensate for the estimated loss-to-follow-up and increase the study power, we increased the sample size in both remdesivir and favipiravir groups to be 106 patients compared to 53 patients in antibodies cocktail group as antibodies cocktail product is available for only about 50 COVID-19 patients. In addition, the ratio (1:2:2) was the closest to reality according to the number of patients who received each drug [11].

The admission rate at Mansoura University – Isolation Hospital was 250 cases per month on average; our needed sample was about 250 cases.

## 7 Results

After statistical analysis using SPSS software, all continuous data showed no normal distribution. So Kruskal–Wallis test was used to compare abnormally distributed continuous, categorical, and nominal variables between the three groups [11].

### 7.1 Regarding baseline characteristics

Table 2 shows the significance of difference between the three groups and also includes a pairwise comparison between every two groups in baseline characteristics if they show a statistically significant difference between the three groups Figures S1–S9 represent distributions and frequencies of baseline characteristics between the three groups [11].

**Table 2:** Significance of differences in baseline characteristics between the three groups

#### 7.1.1 Age

There is a statistically significant difference between A–C and B–C and a statistically non-significant difference between A–B [11].

#### 7.1.2 Gender

There is a statistically significant difference between B–C and a statistically non-significant difference between A–B and A–C [11].

#### 7.1.3 Number of comorbidities

There is a statistically significant difference between B–C and a statistically non-significant difference between A–B and A–C [11].

#### 7.1.4 Method of diagnosis

There is a statistically non-significant difference between the three groups [11].

#### 7.1.5 Severity of COVID-19

There is a statistically significant difference between A–B and A–C and a statistically non-significant difference between C-B. There are statistically significantly less severe cases in group A than in groups B and C [11].

#### 7.1.6 Number of symptoms

There is a statistically significant difference between A–B and A–C and a statistically non-significant difference between C–B [11].

The article "Study to compare the effect of casirivimab and imdevimab, remdesivir, and favipiravir on progression and multi-organ function of hospitalized COVID-19 patients" was retracted in 2023. Reasons: duplicate publication; overlap with earlier publications.

#### 7.1.7 WHO clinical progression scale

There is a statistically significant difference between A–B and A–C and a statistically non-significant difference between C–B. WHO scale is statistically significantly lower in group A than groups B and C.

#### 7.1.8 Multi-organ functions assessment

There is a statistically significant difference between the three groups in SOFA score.

### 7.2 Regression analysis

Regression analysis was performed to explore the effect of baseline characteristics (that show a statistically significant difference between the three groups) on the outcomes of the study and the possibility of existence of confounding variables as shown in Table 3 [11].

**Table 3:** Best regression model for studying effects of confounding variables on WHO scale score

	Unstandardized coefficients		Standardized coefficients		*t*	*P*-value
	*β*	Std. error	*β*	Std. error		
(Constant)	0.806	1.297			0.621	0.535
Age	0.003	0.001	0.098	0.053	1.835	0.78
Gender	0.029	0.044	0.038	0.058	0.652	0.56
Number of co-morbidities	–0.002	0.015	–0.007	0.048	–0.144	0.978
Severity of COVID	–0.004	0.036	–0.007	0.059	–0.123	0.154
WHO clinical progression score	0.024	0.084	0.021	0.071	0.288	0.812
Number of symptoms	0.029	0.033	0.049	0.057	0.854	0.47
SOFA^(1)^	0.012	0.018	0.050	0.077	0.650	0.412

*P-value less than 0.05 is considered a statistically significant difference ^(1)^ Sequential Organ Function Assessment.

### 7.3 Regarding outcomes of the study after intervention in the three groups

Table 4 shows the significance of difference between the three groups and also includes a pairwise comparison between every two groups in clinical outcomes if they show a statistically significant difference between the three groups. Figures S10–S22 in the Supporting Information show the distributions and frequencies of these outcomes across the three groups [11].

**Table 4:** Significance of differences in outcomes between the three groups

#### 7.3.1 Effect on score of multi-organ functions

There is a statistically significant difference in SOFA score on day 3 between the three groups and on days 7 and 14 between A–B and A–C and there are no other statistically significant differences between the groups were observed.

#### 7.3.2 Effect on WHO scale for COVID cases

There is a statistically significant difference in WHO scale on days 3 and 7 between A–B and A–C and on day 14 between A–B only.

For more statistical analysis that is performed on the clinical data of this study, this is a link to a SPSS output file that contains all the statistical analysis of the study. An excel data sheet and a SPSS data file containing all clinical data of the cases of the three groups can be found in the below link in addition to an excel data sheet for included and excluded cases with date [11]: https://drive.google.com/drive/folders/1X1dDQwW9vBvusutwMbeebUjN8jJqYxsh? usp=sharing.

The article "Study to compare the effect of casirivimab and imdevimab, remdesivir, and favipiravir on progression and multi-organ function of hospitalized COVID-19 patients" was retracted in 2023. Reasons: duplicate publication; overlap with earlier publications.

## 8 Discussion

This study compared casirivimab and imdevimab with remdesivir and favipiravir for use in COVID-19 hospitalized patients. There are no similar treatment comparison or related studies to be compared with this research for similarity and differences [11].

### 8.1 Regarding baseline characteristics

The patients’ ages in groups A and B were statistically significantly lower than that in group C. There were statistically significantly more females in group B than group C. The number of co-morbidities is statistically significantly more in group C than Group B. There are statistically significantly less severe cases in group A than groups B and C. There are statistically significantly a smaller number of symptoms in group A than groups B and C. The who scale is statistically significantly lower in group A than groups B and C. Also, SOFA score is higher in group C than groups A and B and in group B than group A. So, A > B > C in multi-organ functions (multi-organ functions were better in A than in B and in B than in C)

### 8.2 Regression analysis

After statistical analysis of baseline characteristics of the cases in the three groups and finding that statistically significant differences in some baseline characteristics existed between the three groups, differences existed between age, gender, number of symptoms, number of co-morbidities, severity of COVID, WHO clinical progression scale, and SOFA score [11].

So, it was necessary to exclude the effect of these variables on the outcomes of the study which was represented by WHO scale score.

For this reason, regression analysis was performed to explore the effects of these variables on the WHO scale score.

After regression analysis, it was found that all baseline characteristics that differed between the three groups had no effect on the study outcome [11].

### 8.3 Regarding outcomes of the study after intervention in the three groups

SOFA score on day 3 was statistically significantly higher in group C than groups A and B and in group B than group A, SOFA score on days 7 and 14 was statistically significantly lower in group A than groups B and C. From these results, it is concluded that the best multi-organ functions are A > B > C with group A having the best multi-organ functions (lowest SOFA score).

Group A has a statistically significantly lower WHO progression scale than Groups B and C on days 3 and 7 and a statistically significantly lower WHO progression scale than Group B on day 14 that proves that less progression of the cases in Group A (lower WHO scale) than Groups B and C.

The article "Study to compare the effect of casirivimab and imdevimab, remdesivir, and favipiravir on progression and multi-organ function of hospitalized COVID-19 patients" was retracted in 2023. Reasons: duplicate publication; overlap with earlier publications.

**Limitations of this study** includes non-randomization of antiviral drugs among included patients, non-blinding of interventions to investigators, applicable only on hospitalized COVID-19 patients (not including outpatients), and the differences in some baseline characteristics between the groups [11].

#### 8.3.1 Generalizations of this study

This study can be generalized on hospitalized COVID-19 patients only and not involve all COVID-19 patients [11].

## 9 Conclusion

Casirivimab and imdevimab achieve less case progression as presented by lower WHO scale and better multi-organ functions as presented by lower SOFA score than remdesivir and favipiravir groups.

From the results, it is observed that Group A (casirivimab and imdevimab) provides better outcomes than groups B (remdesivir) and C (favipiravir).

This research is a long study as posted in the preprint because it contains several outcomes to investigate efficacy and safety of the casirivimab and imdevimab and the other two antiviral agents, so this research is divided into five parts (all parts of the same introduction, methods, patients, and interventions) and will be published in five stages as described in the study protocol due to size limitation in journal publishing. So, this part of the research is an extension of a recently published research paper that was prepared by the same authors. Clinical study to compare the efficacy and safety of casirivimab and imdevimab, remdesivir, and favipiravir in hospitalized COVID-19 patients that has been cited in the manuscript (reference no: 11) is available in the following links:https://doi.org/10.1016/j.jcvp.2023.100151, https://www.ncbi.nlm.nih.gov/pmc/articles/PMC10169321/, https://www.sciencedirect.com/science/article/pii/S2667038023000182?via%3Dihub Preprints for this study are available at two websites. Clinical study to evaluate the possible efficacy and safety of antibodies combination (casirivimab and imdevimab) vs standard antiviral therapy as antiviral agent against coronavirus-2 infection in hospitalized COVID-19 patients is available in the following links: https://www.medrxiv.org/content/10.1101/2022.08.20.22279020v2.full.pdf, https://www.researchsquare.com/article/rs-1991618/v2. For more statistical analysis that is performed on clinical data of this study, below is the link to an SPSS output file that contains all the statistical analysis of the study. An excel data sheet and an SPSS data file containing all clinical data of the cases of the three groups can be found in this link in addition to an excel data sheet for included and excluded cases with date: https://drive.google.com/drive/folders/1X1dDQwW9vBvusutwMbeebUjN8jJqYxsh? usp=sharing,

The article "Study to compare the effect of casirivimab and imdevimab, remdesivir, and favipiravir on progression and multi-organ function of hospitalized COVID-19 patients" was retracted in 2023. Reasons: duplicate publication; overlap with earlier publications.

## Supplementary Material

Supplementary Figure
